# Biomechanical Effect of Valgus Knee Braces on the Treatment of Medial Gonarthrosis: A Systematic Review

**DOI:** 10.1155/2022/4194472

**Published:** 2022-05-29

**Authors:** Yuzhou Yan, Geng Liu, Li Zhang, Ruitao Gong, Pengge Fu, Bing Han, Hui Li

**Affiliations:** ^1^Innovation Center of Bioengineering, Shaanxi Engineering Laboratory for Transmissions and Controls, Northwestern Polytechnical University, Xi'an 710072, China; ^2^Joint Surgery Department, Xi'an Hong-Hui Hospital, Xi'an Jiaotong University College of Medicine, Xi'an 710054, China

## Abstract

**Background:**

Valgus braces are prescribed as a common conservative treatment option for patients with medial gonarthrosis to improve their quality of life. Many studies had reviewed the effects of the valgus braces on patients with medial gonarthrosis, while they mainly focused on the knee adduction moment (KAM), with less attention paid to other parameters such as spatiotemporal and morphological parameters.

**Objectives:**

The purpose of this study was to review the effects of valgus braces on the spatiotemporal, kinematic/kinetic, morphological, and muscle parameters.

**Methods:**

Based on the selected keywords, a survey of literatures was performed in Web of Science, PubMed, Scopus, and Google Scholar using the PRISMA methods, and the search period was established from January 2000 to March 2022.

**Results:**

Thirty-four articles were included. According to the conclusion of these articles, the valgus brace can be used to relieve the symptoms of patients with medial gonarthrosis by decreasing the varus angle, decreasing the KAM, and redistributing the knee compartment loads. However, the effects of valgus braces on other biomechanical parameters (e.g., walking speed, cadence, joint angle, and joint space) had not reached a consensus.

**Conclusions:**

The valgus knee brace can effectively relieve the symptoms of medial gonarthrosis through multiple mechanisms, while there is still some confusion about the effectiveness of the valgus brace on the other biomechanical parameters.

## 1. Introduction

Gonarthrosis is a widespread degenerative musculoskeletal disease that typically occurs in elderly people, obese people, and those who have suffered from a lower limb injury [1, 2]. Due to the physiological geometry of the tibial plane, the internal forces of the knee show nonuniform distribution in the tibial plane during motion [3]. Generally, 60-80% of the compressive load transmitted throughout the knee is applied on the medial compartment, which means that the loads on medial compartment are approximately 2.2 times higher than the lateral compartment [4]. Therefore, there will be more severe effects of gonarthrosis on the medial compartment compared with the lateral compartment [5].

Varus alignment may be a cause or result of gonarthrosis, which will result in the overload of medial compartment and cartilage wear [6, 7]. If the intervention and therapy are not taken, the total knee arthroplasty (TKA) will be the only option due to the deterioration of gonarthrosis. Unfortunately, doctors only advise TKA to patients with severe gonarthrosis due to the invasive nature of the surgery, the high costs, and the risk of complications [4]. Approximately 19% of TKA patients are unsatisfied with their treatment, especially those under the age of 70, who met a higher risk of renovation surgery [8].

Currently, the valgus knee brace, a common and effective conservative treatment option, has been shown to be effective in delaying the progression of the medial gonarthrosis. The valgus knee brace improves the knee joint alignment by applying an auxiliary force in the coronal plane, and the load will be transferred to the lateral compartment. Then, the contact forces on the medial compartment were decreased, and the suffering of the patients could be relieved [9, 10].

In the past few decades, the treatment effects of valgus braces on medial gonarthrosis have been reviewed in several related studies. Ramsey and Russell [11] summarized the effects of valgus braces on kinematic/kinetic and perception parameters, and the joint space, joint moment, and joint load were analyzed. Alfatafta H et al. [12] and Khosravi et al. [13] reviewed the effects of valgus braces on pain and functional activity levels of patients with medial gonarthrosis, while the biomechanical effects of valgus braces were excluded in this paper. Moyer et al. [14] assessed the biomechanical effects of braces on medial gonarthrosis, which focused on the knee joint moment, joint space, and muscle cocontraction. The effects of valgus braces on spatiotemporal and kinematic parameters were not involved. Petersen et al. [15] evaluated the biomechanical effects of valgus braces on medial gonarthrosis, which included the effects on the knee adduction moment (KAM). Steadman et al. [16] reported the effects of valgus braces on clinical application and biomechanical parameters such as joint load, joint space, and varus angle. Overall, most studies have concentrated on the effects of braces on KAM and pain index, with little attention paid to other parameters. The KAM and ache index may reflect the effect of braces on patients with medial gonarthrosis, while some studies have proven that the real situation of the knee compartment can be reflected by the KAM partially [17–19], so other parameters such as spatiotemporal, kinematic/kinetic, morphological, and muscle parameters should be considered to further understand the effects of valgus braces on medial gonarthrosis.

Therefore, the purpose of this review article is to critically evaluate the biomechanical effects of the valgus knee braces on patients with medial gonarthrosis such as spatiotemporal, kinematic/kinetic, and morphological parameters. This review would help understand the biomechanical effects of valgus braces and possibly improve their design and effectiveness.

## 2. Methods

This review followed the Preferred Reporting Items for Systematic Review and Meta-Analyses (PRISMA) guidelines [20].

### 2.1. Search Strategy

In this paper, three online databases (Web of Science, PubMed, and Scopus) were searched by 3 independent reviewers in triplicate for relevant articles from January 1, 2000, to March 1, 2022. Search terms such as “unloader brace”, “valgus brace”, “medial compartment knee osteoarthritis”, “medial gonarthrosis”, and “knee orthosis” were used. A manual search of included papers' references and abstracts from recent conferences, as well as Google Scholar, was conducted to find any further related research.

### 2.2. Assessment of Study Eligibility

The inclusion and exclusion criteria were determined ahead of time. The following criteria were used to determine eligibility: (1) the treatment of medial gonarthrosis, (2) at least one knee brace, and (3) biomechanical evaluation of knee braces. Exclusion criteria included (1) nonhuman studies, (2) other types of orthoses instead of knee valgus brace, (3) other pathological conditions, (4) studies involving the effect of orthotic devices on other knee disorders, (5) pain or activity level outcome using Western Ontario and McMaster Universities Osteoarthritis Index (WOMAC), 36-item Short-form Health Survey (SF-36), Knee Injury and Osteoarthritis Outcome Score (KOOS), Visual Analog Scales (VAS), etc., and (6) systematic reviews or meta-analyses. If an article contained both biomechanical and clinical results, the article would be retained, and only the biomechanical results were analyzed.

### 2.3. Study Screening

Three reviewers (YZY, LZ, and RTG) independently screened all titles, abstracts, and full-text articles. Any discrepancies at the title and abstract stages were tolerated, and the articles were forwarded to the next step of screening to ensure that relevant articles were not overlooked. The three reviewers discussed their disagreements at the full-text stage. When they could not reach a consensus, the opinion of the senior reviewer (GL) was considered to determine the eligibility of the article.

## 3. Results

Following the selection procedure, 34 studies that evaluated the effects of valgus braces on medial gonarthrosis were matched the inclusion criteria in this review. The search process is demonstrated using the diagram in Figure 1, and the biomechanical parameters summarized in this review are shown in Figure 2.

### 3.1. Brace Condition

Valgus knee brace, as a common and effective conservative treatment, applies bending moment at the knee joint, modifies the knee joint alignment in the coronal plane, shifts the load from the medial compartment to the lateral compartment, and reduces the forces in the medial compartment. The use of different types of valgus braces has been reported to delay the deterioration of the medial gonarthrosis and reduce knee pain. The traditional valgus brace currently on the market could be divided into two types, single-hinged and double-hinged, as shown in Figures 3(a) and 3(b). In recent years, researchers optimized the braces to make patients feel comfortable, mainly by adding the air cushion (Figure 3(c)), increasing the freedom of the brace (Figure 3(d)), and introducing the control systems (Figure 3(e)). The 34 articles included in this article contained 19 different types of knee valgus braces, including 7 types of single-hinged braces, 6 types of double-hinged braces, and 6 types of modified braces (3 with air cushions, 2 with structural optimization, and 2 with control system).

### 3.2. Spatiotemporal Parameters

As shown in Table 1, the spatiotemporal parameters reviewed in this review included walking speed, cadence, step length and stride length, stride width, and foot progression angle (FPA). The variations of spatiotemporal parameters between the braced and unbraced conditions are shown in Table 2.

#### 3.2.1. Walking Speed

Eight studies found that the use of a knee valgus brace significantly improved walking speed, with a maximum increase of 23.53% and a minimum increase of 4.32% [26, 30–32, 35, 36, 38, 39]. However, seven studies reported no significant difference in walking speed when patients wore the brace [21, 27–29, 33, 34, 37], and two of those studies even showed negative effects of valgus braces on walking speed [29, 33].

#### 3.2.2. Cadence

The number of steps taken per minute is called the cadence, also known as the step rate [40]. Four studies discussed the effects of valgus braces on cadence. Two studies found that cadence was significantly raised after wearing the brace, with an increase of 2.80% [38] and 4.40% [39], respectively. However, two studies showed no statistical difference between braced and unbraced conditions [27, 33].

#### 3.2.3. Step Length and Stride Length

The distance in one step is called the step length, and the distance between two consecutive heel contacts of the same foot is called the stride length [40], as described in Figure 4. Three studies found that the valgus braces were effective in improving step length and stride length in the arthritic limb, with a maximum increase of 16.90% and a minimum increase of 5.66% [26, 30, 38], as shown in Table 2, whereas six studies showed that the braces had no significant improvement in step length and stride length [27, 33, 34, 39] and even had a negative effect on step length due to the restriction of range of motion (ROM) in the sagittal plane [21, 31].

#### 3.2.4. Step Width

As shown in Figure 4, the distance between the centers of heels of two consecutive feet touching each other is called the step width [40]. Despite two studies reported the change in step length, there was no statistical difference in either study [21, 36], as shown in Table 2. But Laroche et al. [36] discovered that the stride width of the two limbs tended to be constant after wearing a brace.

#### 3.2.5. FPA

The angle generated between the longitudinal axis of the foot and the forward line of progression when walking is known as the FPA [40, 41], which has been associated with the KAM and might be used to reduce joint loading and pain [42–45]. Laroche et al. [36] revealed that the FPA increased by an average of 36.76% after wearing a brace. However, Brand et al. and Gaasbeek et al. found no significant difference in FPA compared to the unbraced condition [27, 31].

### 3.3. Kinematic and Kinetic Parameters

Currently, researchers have focused on the biomechanical effects of valgus braces, especially whether the kinematic and kinetic parameters changed after the patients wearing the brace, as shown in Table 3.

#### 3.3.1. Knee Joint Angle

The knee joint angle could be divided into the flexion-extension angle (sagittal plane) and the adduction-abduction angle (frontal plane), as shown in Figure 5(a). The effects of valgus braces on knee joint angle were investigated in five studies. Laroche et al. [36] discovered that the knee extension angle at heel strike (HS) and midstance (MS) was significantly increased after wearing the brace. Brand et al. [27] indicated that the knee adduction angle in braced condition was decreased by 84.31% and 55.31% at HS and push-off (PO), respectively. Toriyama et al. [39] found that only the contralateral knee adduction angle was significantly increased by an average of 0.32° during 46%-55% of the stance phase in the braced condition. Two studies showed that the flexion-extension angle did not significantly change during the gait [29, 49].

#### 3.3.2. Knee Range of Motion

Knee ROM is mainly represented as the range of flexion/extension angles during knee movement, as shown in Figure 5(a). Four studies investigated the effects of valgus braces on the knee ROM. Arazpour et al. [26] discovered that knee ROM was decreased by 11.36% after wearing the brace. Fesharaki et al. [30] found a maximum reduction of 25.68% in knee ROM with wearing the brace. Gaasbeek et al. [31] reported that the brace significantly decreased the ROM by 5.45%. However, one study [33] found no significant difference in knee ROM between braced and unbraced conditions.

#### 3.3.3. Ground Reaction Force (GRF) and Foot Pressure

Four studies reported the effects of valgus braces on GRF (Figure 5(b)). Three studies found no significant difference between braced and unbraced conditions [27, 33, 52]. However, Schmalz et al. [38] argued that the horizontal force on the arthritic limb was increased by 16.4% BW in brace condition. One study observed the changes in foot pressure. Kim et al. [50] found that the lateral-side foot pressure was significantly reduced during the stance phase.

#### 3.3.4. Knee Joint Moment

Knee joint moment included knee adduction moment (KAM) and knee flexion moment (KFM), as shown in Figure 5(c). Seventeen studies evaluated the effects of valgus braces on the KAM, and nine studies reported the change of the mean KAM [21, 22, 26, 28, 29, 32, 37, 46, 54], while nine studies reported the change of the first and second peak KAM separately [24, 27, 31, 35, 36, 39, 47, 48, 54]. Most studies showed that the braces significantly reduced the KAM, with a maximum reduction of 48% and a minimum reduction of 3.63%. But two studies found no significant difference in the KAM [22, 46], as shown in Table 4. Meanwhile, two studies showed a significant trend of improvement in the KFM [21, 39].

#### 3.3.5. Knee Adduction Moment Impulse (KAI)

KAI, which considers both the magnitude and duration of stance, is more sensitive at differentiating between disease severities and may provide a more comprehensive description of medial knee joint load [56, 57], as shown in Figure 5(d). Three studies indicated that braces were effective in reducing KAI. Fantini et al. [47, 48] discovered a maximum reduction in KAI of 36% when the brace set to 8° valgus mode. Lamberg et al. [35] demonstrated that the KAI in the second half of the stance phase was significantly decreased by 36%. However, Laroche et al. [36] held an opposite view, and they reported that KAI did not show any significant difference.

#### 3.3.6. Knee Contact Forces and Stress

The KAM was considered to be a surrogate measure of knee contact force (KCF), while researchers discovered a moderate correlation between KAM and KCF [58–60]. To better understand the effects of valgus brace on the knee compartment, the researchers calculated KCF and cartilage stresses through musculoskeletal models, and the typical results are shown in Figure 5(e). Six studies reported the changes in KCF. Four studies reported that the medial knee compartment contact force (MKCF) was significantly reduced in brace condition [22, 34, 37, 49], indicating that the load was shifted to lateral compartment. Two studies discovered no significant difference in the peak KCF between the braced and unbraced conditions [21, 33]. Three publications mentioned the change of contact stress by using the finite element method. Two studies confirmed that the brace significantly reduced the peak contact stress in the medial compartment while increased in the lateral compartment [51, 55]. One study [53] showed that the mean contact stress and contact area of the medial compartment were not changed when the knee joint was at 5-10° and 15-20° flexion states.

#### 3.3.7. Interactive Force

The interactive force could be divided into the valgus force, brace abduction moment (BAM), and shear force. The shear force is commonly generated at the interface between the brace and the thigh. Six publications evaluated the interactivity force between the brace and the human body. One study reported a maximum valgus force of 60 N, which was maintained constant throughout the stance phase [54]. Three studies described the BAM, which was around 10% of the KAM, and suggested that BAM was associated with valgus angulations or strap tensions [25, 37, 38]. Two studies mentioned that the 2 degree-of-freedom (DOF) brace decreased the external shear force by 41.31 ± 8.34 N compared to the 1-DOF brace when knee joint at 90° flexion states [24, 30], as shown in Figure 5(f).

### 3.4. Morphological Parameters

Lower limb malalignment, dynamic knee joint space, and medial cartilage cross-sectional area (MCCA) are the morphological parameters of interest to researchers, as shown in Table 5.

#### 3.4.1. Lower Limb Malalignment

Lower limb malalignment is presumed to cause and/or accelerate gonarthrosis, which is usually denoted by the knee varus angle (Figure 6(a)) [7, 65–67]. Two studies used anterior/posterior X-rays to observe lower limb malalignment under static standing conditions. Arazpour et al. [23] found that the varus angle was decreased by 6° when the patient wore the brace. Draganich et al. [29] reported that the knee varus angle was decreased by an average of 1.5° after wearing the bespoke brace.

#### 3.4.2. Dynamic Knee Joint Space

To understand the effects of valgus braces on the knee joint space during walking, the researchers used biplane radiographs or three-dimensional (3D) fluoroscopy methods to analyze the dynamic changes in the knee joint space [68, 69], as shown in Figure 6(b). Four studies revealed the effects of valgus braces on the treatment of gonarthrosis. Dennis et al. [61] reported that the medial compartment separation increased by an average of 1.3 mm during the gait cycle. Dessinger et al. [62] found that 80% of patients experienced a medial joint space increase of more than 1.0 mm at heel strike, while 65% had a similar change during midstance. Nagai et al. [52] showed that the dynamic space of the medial compartment was significantly increased by 0.3 mm after wearing the brace. In addition, one study [63] found no significant difference in the separation of the medial and lateral compartments between the braced and unbraced conditions.

#### 3.4.3. MCCA

The articular cartilage response to loading is dependent on the magnitude and rate of the load [70, 71], so observing the deformation of MCCA by ultrasonic testing techniques can be used to evaluate the effects of valgus braces, as shown in Figure 6(c). In 2019, Pfeiffer et al. [64] showed no significant difference in percent change of MCCA between the braced and unbraced conditions.

### 3.5. Muscle Parameters

Only five (of 34) studies examined the effects of valgus braces on muscle parameters such as muscle activation, muscle strength, relative contribution of muscle, and cocontraction ratios (CCRs), as shown in Table 6. Brandon et al. [22] reported that only the electromyography (EMG) of the biceps femoris was significantly reduced during walking after wearing the brace, as shown in Figure 7(a). Fantini et al. [72] found that the muscle activation and CCRs were significantly reduced in all muscle groups (rectus femoris, lateral hamstring, and gastrocnemius lateralis), but only the 4° valgus mode caused differences in CCRs between the muscle groups. Hall et al. [21] found that the peak medial-to-lateral muscle CCRs were reduced and the peak extensor-to-flexor muscle CCRs increased at midlate stance, as shown in Figure 7(b). Total muscle activation and relative contribution of muscles to medial compartment load were not significantly changed compared with the unbraced condition, as shown in Figures 7(c) and 7(d). But the relative contribution of muscles to the lateral compartment was increased by 2.35% after wearing a brace. Thigh girth measurement was used as a biomarker of quadriceps strength by Johnson et al. [32], and patients who satisfied the criteria showed an average increase of 1.90 cm in thigh girth measurement after three months of treatment. Ebert et al. [46] found no significant difference in total muscle activation and the mediolateral-directed CCRs with and without wearing the brace, which might be attributable to the fact that the experimental subjects were healthy individuals.

## 4. Discussion and Conclusions

This systematic review was conducted to evaluate the spatiotemporal, kinematic/kinetic, morphological, and muscle effects of valgus braces on patients with medial gonarthrosis, suggesting that the valgus brace could significantly change the biomechanics of the knee joint during daily activities through a multitude of mechanisms. Studies found that the potential mechanisms of valgus braces included applying valgus moments at the knee to directly oppose KAM [21, 23, 26, 28], altering the alignment of the lower limbs in the frontal plane [23, 29], increasing medial joint space during gait [52, 61, 62], and increasing knee stability to reduce muscle cocontraction [21, 72].

This systematic review showed that the biomechanical effects of valgus braces on patients with gonarthrosis were still contradictory. The contradictory results between the studies might be associated with the differences in the type of braces and the duration of treatment [22, 35, 40, 61] or might also be related to the physiological conditions of the subjects [46, 62]. Most researchers showed that the knee braces could reduce the KAM [26, 29, 32, 35, 36, 47, 48] and KCF [21, 22, 33, 34], while other biomechanical parameters were not significantly changed. Even though KAM and KCF were closely related to the progression of gonarthrosis, they did not cause gonarthrosis alone. Therefore, the effects of valgus braces on biomechanical parameters should be fully considered in future studies.

Some limitations of the current studies must be noted. First, the knee ROM is significantly recued, which might lead to a reduction in foot clearance and a shorter step length [26, 30, 31]. Second, few studies evaluate the patient compliance. Studies reported that patient compliance reduced as the duration of treatment increased, which might affect the real treatment effects of valgus braces [73, 74]. Third, the quantitative relationship between the valgus angle and the KCF is not established. The valgus force was empirically adjusted to the level of comfort accepted by the patients, which may lead to different treatment effects on different patients. Fourth, the long-term biomechanical effects of valgus braces are not studied. The valgus braces must be used for several years as a conservative treatment for gonarthrosis. The load transferred to the lateral compartment by the valgus braces might aggravate the wear of lateral cartilage, which might have negative effects in the long term [16, 22].

This review still has some limitations. First, only studies published in English were included, which created a language bias in the selection of articles. Second, the review findings are limited to the studies identified by the set search strategy. Third, we were unable to pool data in the form of a meta-analysis because of the heterogeneity of the outcome measure and the various comparison groups used in the included studies.

In conclusion, this review showed that the valgus knee brace can effectively improve the symptoms of medial gonarthrosis through multiple mechanisms, primarily by decreasing the varus angle, reducing the KAM, and redistributing the knee compartment loads. However, the current studies suggested that the effects of valgus braces on other biomechanical parameters were still controversial.

## Figures and Tables

**Figure 1:** The PRISMA flow diagram of the study selection process.

**Figure 2:** Tree diagram displaying the investigated biomechanical parameters. GRF: ground reaction force; KAI: knee adduction moment impulse.

**Figure 3:** Typical structures of the valgus knee brace. (a) Single-hinged valgus brace (Ossür Unloader One® brace [21]). (b) Double-hinged valgus brace (OA Adjuster brace [22]). (c) Brace with two air cushions [23]. (d) Brace with two degree-of-freedom (DOF) [24]. (e) Brace with control system [25].

**Figure 4:** Spatial description of gait. FPA: foot progression angle.

**Figure 5:** Kinematic and kinetic description of gait. (a) Knee joint angle and knee range of motion (ROM). (b) Ground reaction force [38]. (c) Knee adduction moment (KAM) and flexion moment (KFM). (d) Knee adduction moment impulse (KAI). (e) Knee joint contact force [21]. (f) Shear force between the brace and human [24], DOF: degree-of-freedom.

**Figure 6:** The morphological parameters of a knee joint. (a) Knee varus angle [23]. (b) Dynamical knee joint space [62]. (c) Ultrasonographic image of the femoral articular cartilage with the medial compartment cross-sectional area [64].

**Figure 7:** Changes in knee joint muscle parameters. (a) Mean enveloped electromyography (EMG) of biceps femoris (BF) in unbraced, OA Adjuster 3, and OA Assist braced condition [22]. (b) Cocontraction ratios (CCRs) with/without brace [21]. (c) Muscle activation with/without brace [21]. (d) Relative contributions of muscle to medial and lateral compartment tibiofemoral contact force with/without brace [21]. M+L: medial and lateral directed; F+E: flexion and extension directed.

**Table 1:** Studies that evaluated the effect of knee brace on spatiotemporal parameters in medial gonarthrosis.

References	Type of brace	Sample size	Duration	Study design	Outcome measurements	Results
Arazpour et al. [26]	Double-hinged brace (air cushions)	7 P (5F/2M)	Immediate effect	Walk	Walking speed Step length	The walking speed and step length were significantly increased.
Brand et al. [27]	Double-hinged brace	22 P (10F/12M)	2 weeks	Walk	Walking speed Step length Cadence FPA	The walking speed, step length, step cadence, and FPA were not significantly changed.
Croce et al. [28]	Single-hinged brace (air cushions)	18 P (6F/12M)	Immediate effect	Walk	Walking speed	The average walking speed was not statistically changed between the unbraced, uninflated, and 7 psi conditions.
Draganich et al. [29]	Double-hinged brace	10 P (-)	4-5 weeks	Walk	Walking speed	The walking speed was not significantly changed.
Fesharaki et al. [30]	Double-hinged brace (two DOF)	16 (11F/5M)	Immediate effect	Walk	Walking speed Stride length	The walking speed and stride length were significantly increased.
Gaasbeek et al. [31]	Single-hinged brace (air cushions)	15 P (3F/12M)	6 weeks	Walk	Walking speed Step length FPA	The walking speed was increased and the step length was reduced. FPA was not significantly changed.
Hall et al. [21]	Single-hinged brace	16 H (7F/9M)	Immediate effect	Walk	Walking speed Stride length Step width	The walking speed, stride length, and stride width were not significantly changed.
Johnson et al. [32]	Double-hinged brace	10 P (4F/6M)	3 months	Walk	Walking speed	The average walking speed increased from 100 cm/s to 112 cm/s.
Karimi et al. [33]	Double-hinged brace	5 P (-)	Immediate effect	Walk	Walking speed Stride length Cadence	The walking speed, stride length, and cadence were not significantly changed.
Kutzner et al. [34]	Single/double-hinged brace	3 P (-)	Immediate effect	Walk	Stride length	The stride length was not significantly changed.
Lamberg et al. [35]	Double-hinged brace	15 P (3F/12M)	2 weeks 8 weeks	Walk	Walking speed	The walking speed was significantly increased.
Laroche et al. [36]	Double-hinged brace	20 P (16F/4M)	5 weeks	Walk	Walking speed Step width FPA	The walking speed was definitely increased. Step width was not statistically changed. FPA was significantly reduced at the TS and PO phase.
Pollo et al. [37]	Single-hinged brace	11 P (-)	>2 weeks	Walk	Walking speed	The walking speed was not significantly changed.
Schmalz et al. [38]	Single-hinged brace	16 P (8F/8M)	4 weeks	Walk	Walking speed Cadence Step length	The mean walking speed, cadence, and step length were significantly increased.
Toriyama et al. [39]	Single-hinged brace	19 P (17F/2M)	Immediate effect	Walk	Walk speed Cadence Step length Stride length	The walking speed and cadence were significantly increased. Other variables were not significantly changed.

P: patient; F: female; M: male; H: healthy; (-): not mentioned; DOF: degree-of-freedom; FPA: foot progression angle; TS: terminal stance; PO: push-off.

**Table 2:** The variations of spatiotemporal parameters between braced and unbraced conditions.

References	Walking speed	Cadence	Step/stride length	Step width	FPA
Arazpour et al. [26]	5.60%	0.00%	5.66%	—	—
Brand et al. [27]	0.00%	0.00%	0.00%	—	0.00%
Croce et al. [28]	0.00%	—	—	—	—
Draganich et al. [29]	-6.67%	—	—	—	—
Fesharaki et al. [30]	23.53%	—	15.48%	—	—
Gaasbeek et al. [31]	5.83%	—	-1.75%	—	0.00%
Hall et al. [21]	0.00%	—	-2.69%	0.00%	—
Johnson et al. [32]	12.00%	—	—	—	—
Karimi et al. [33]	-8.43%	0.00%	0.00%	—	—
Kutzner et al. [34]	0.00%	—	0.00%	—	—
Lamberg et al. [35]	11.11%	—	—	—	—
Laroche et al. [36]	7.14%	—	—	0.00%	36.76%
Pollo et al. [37]	0.00%	—	—	—	—
Schmalz et al. [38]	9.00%	2.80%	16.90%	—	—
Toriyama et al. [39]	4.32%	4.40%	0.00%	—	—

(-): not mentioned; 0.00%: no statistical differences between braced and unbraced conditions. FPA: foot progression angle.

**Table 3:** Studies that evaluated the effect of knee brace on kinetic and kinematic parameters in medial gonarthrosis.

References	Type of brace	Sample size	Duration	Study design	Outcome measurements	Results
Arazpour et al. [26]	Double-hinged brace (air cushions)	7 P (5F/2M)	Immediate effect	Walk	KAM ROM	The KAM was significantly reduced. Knee ROM in sagittal plane was significantly decreased.
Brand et al. [27]	Double-hinged brace	22 P (10F/12M)	2 weeks	Walk	KAM GRF Joint angle	The KAM and knee adduction angle were significantly reduced. The GRF was not significantly changed.
Brandon et al. [22]	Single/double-hinged brace	17 P (8F/9M)	Immediate effect	Walk	KAM Contact force	The KAM was not significantly changed unless the brace moment was included. The medial compartment load was significantly reduced.
Croce et al. [28]	Single-hinged brace (air cushions)	18 P (6F/12M)	Immediate effect	Walk	KAM	The KAM decreased by 7.6% with the air cushion uninflated and decreased by 26.0% with the air cushion inflated to 7 psi.
Draganich et al. [29]	Double-hinged brace	10 P (-)	4-5 weeks	Walk	KAM Joint angle	The KAM was significantly reduced. The knee flexion angle was not significantly changed.
Ebert et al. [46]	Double-hinged brace	20 H (10F/10M)	Immediate effect	Walk	KAM	The KAM was not significantly changed.
Fantini et al. [47]	Single-hinged brace	16 H (-)	Immediate effect	Walk	KAM KAI	The KAM was reduced during walking and running tasks. The KAI of 4° and 8° valgus mode were decreased by 25% and 36%, respectively.
Fantini et al. [48]	Single-hinged brace	11 P (8F/3M)	2 weeks	Walk	KAM KAI	The KAM was significantly reduced. Changes in KAI of 4° valgus and flexible adjustable were 29% and 15%, respectively.
Fesharaki et al. [30]	Double-hinged brace (two-DOF)	16 P (11F/5M)	Immediate effect	Walk Sit-stand-sit	KAM ROM Shear force	The KAM was significantly reduced in walking. In the sit-to-stand test, the knee ROM was significantly reduced, and the shear force was decreased by 41.31 ± 8.34 N.
Fesharaki et al. [24]	Double-hinged brace (two-DOF)	1 P (1M)	Immediate effect	Sit-stand-sit	Shear force	The shear force was decreased by 45 N.
Gaasbeek et al. [31]	Single-hinged brace (air cushions)	15 P (3F/12M)	6 weeks	Walk	KAM ROM	The KAM and ROM was significantly reduced.
Hall et al. [21]	Single-hinged brace	16 H (7F/9M)	Immediate effect	Walk	Contact force KFM KAM	The medial compartment load was not significantly changed. The KFM and KAM were significantly reduced.
Huber et al. [49]	Double-hinged brace	2 H (-)	Immediate effect	Walk	Joint load Brace force Joint angle	The knee loads were significantly reduced. The device provided a supportive moment during stance. The knee extension angle was not changed.
Johnson et al. [32]	Double-hinged brace	10 P (4F/6M)	3 months	Walk	KAM	The KAM was decreased by 0.23 Nm/kg.
Karimi et al. [33]	Double-hinged brace	5 P (-)	Immediate effect	Walk	Contact force ROM GRF	The mean values of peak knee contact force in the vertical and mediolateral directions, knee ROM, and GRF were not statistically changed.
Kim et al. [50]	Single-hinged brace (control system)	3 H (3M)	Immediate effect	Walk	Foot pressure	The lateral-side foot pressure was significantly reduced during the stance phase.
Kutzner et al. [34]	Single/double-hinged brace	3 P (-)	Immediate effect	Walk	Contact force	The medial forces were significantly reduced during walking, while the medial forces were reduced only with the MOS brace during ascending or descending stairs.
Lamberg et al. [35]	Double-hinged brace	15 P (3F/12M)	2 weeks 8 weeks	Walk	KAI KAM Joint angle	The KAI and KAM were significantly reduced. The peak knee extension angle during the stance phase was decreased.
Laroche et al. [36]	Double-hinged brace	20 P (16F/4M)	5 weeks	Walk	KAM Joint angle KAI	The KAM was significantly reduced at the TS and PO phase. The knee internal/external rotation angle and KAI did not show any significant difference.
Marius et al. [51]	Double-hinged brace	—	—	Simulation analysis	Contact stress	The femoral cartilage stress, tibia cartilage stress, and menisci stress were significantly reduced.
Nagai et al. [52]	Double-hinged brace	10 P (2F/8M)	2 weeks	Walk	GRF	The vertical compartment of GRF was not significantly changed.
Pollo et al. [37]	Single-hinged brace	11 P (-)	>2 weeks	Walk	KAM BAM Joint loads	The KAM and the medial compartment load were significantly decreased by 13% and 11%, respectively. The maximum BAM was 11.0 Nm when the brace set to 8° valgus mode.
Reinsdorf et al. [25]	Single-hinged brace (control system)	1 H (-)	Immediate effect	Walk	BAM	The peak BAM was 8.7 Nm, and the maximum raise of BAM was 37 Nm/s during 0-15% GC.
Schmalz et al. [38]	Single-hinged brace	16 P (8F/8M)	4 weeks	Walk	BAM GRF	The maximum BAM was 0.05 Nm/kg, which represents approximately 10% of the natural KAM. The vertical compartment of the GRF was decreased, but the horizontal force was increased by 16.4% BW.
Segal et al. [53]	Single-hinged brace	15 P (9F/6M)	Immediate effect	Static standing	Contact stress Contact area	The mean contact stress and contact area of the medial compartment were not significantly changed during the 5°–10° and 15°-20° flexion conditions.
Self et al. [54]	Single-hinged brace	5 P (1F/4M)	2 weeks	Walk	KAM Brace force	The KAM was significantly reduced at 20% and 25% of stance phase. The valgus force remained constant throughout the first 80% of the stance phase.
Shriram et al. [55]	—	1 H (1M)	—	Walk	Contact force Contact area	The total contact force, contact area, and contact pressure of the medial and lateral compartment were significantly changed.
Toriyama et al. [39]	Single-hinged brace	19 P (17F/2M)	Immediate effect	Walk	KAM KFM Joint angle	The KFM and KAM were significantly reduced. During 46%-55% of the stance phase, the knee adduction angle was significantly increased by an average of 0.32°.

P: patient; F: female; M: male; H: healthy; (-): not mentioned; GC: gait cycle; BW: body weight; GRF: ground reaction force; DOF: degree-of-freedom; KAM: knee adduction moment; KFM: knee flexion moment; KAI: knee adduction impulse; TS: terminal stance; PO: push-off; BAM: brace abduction moment.

**Table 4:** The maximum change of KAM between braced and unbraced condition.

References	First peak of KAM	Second peak of KAM	Mean KAM	KFM
Arazpour et al. [26]	—	—	3.63%	—
Brand et al. [27]	18.55%	17.00%	—	—
Brandon et al. [22]	—	—	0.00%	—
Croce et al. [28]	—	—	24.39%	—
Draganich et al. [29]	—	—	6.90%	—
Ebert et al. [46]	—	—	0.00%	—
Fantini et al. [47]	0.00%	33.89%	—	—
Fantini et al. [48]	0.00%	16.66%	—	—
Fesharaki et al. [24]	10.83%	9.80%	—	—
Gaasbeek et al. [31]	11.52%	14.63%	—	—
Hall et al. [21]	—	—	10.71%	10.96%
Johnson et al. [32]	—	—	48.00%	—
Lamberg et al. [35]	15.87%	25.00%	—	—
Laroche et al. [36]	26.10%	21.92%	—	—
Pollo et al. [37]	—	—	7.59%	—
Self et al. [54]	11.82%	0.00%	25.00%	—
Toriyama et al. [39]	11.10%	0.00%	—	142.90%

(-): not mentioned; 0.00%: no statistical differences between braced and unbraced conditions; KAM: knee adduction moment; KFM: knee flexion moment.

**Table 5:** Studies that evaluated the effect of knee brace on morphological results in medial gonarthrosis.

References	Type of brace	Sample size	Duration	Study design	Outcome measurements	Results
Arazpour et al. [23]	Double-hinged brace (air cushions)	1 P (1F)	Immediate effect	Static standing	Varus angle	The knee varus rotation angle was reduced by 6°.
Dennis et al. [61]	Double-hinged brace	45 P (-)	Immediate effect	Walk	DJS	78% of patients at heel strike and 70% of patients at midstance phase were observed medial condylar separation.
Dessinger et al. [62]	Single-hinged brace	20 P (-)	Immediate effect	Walk	DJS	The medial joint space was significantly increased, and the location of the contact point was lateral shifted.
Draganich et al. [29]	Double-hinged brace	10 P (-)	4-5 weeks	Static standing	Varus angle	The knee varus angle was significantly decreased by 1.5°.
Haladik et al. [63]	Double-hinged brace	10 P (1F/9M)	2 weeks	Walk	DJS	The joint space and contact center location were not significantly changed.
Nagai et al. [52]	Double-hinged brace	10 P (2F/8M)	2 weeks	Walk	DJS	Medical compartment DJS was significantly increased.
Pfeiffer et al. [64]	—	24 H (15F/9M)	1 week	Walk	MCCA	The percent change of MCCA was no different.

P: patient; F: female; M: male; H: healthy; (-): not mentioned; DJS: dynamic joint space; MCCA: medial cartilage cross-sectional area.

**Table 6:** Studies that evaluated the effect of knee brace on muscle in medial gonarthrosis.

References	Description of brace	Sample size	Duration	Study design	Outcome measurements	Results
Brandon et al. [22]	Single/double-hinged brace	17 P (8F/9M)	Immediate effect	Walk	EMG	Only the EMG of the biceps femoris was significantly reduced.
Ebert et al. [46]	Double-hinged brace	20 H (10F/10M)	Immediate effect	Walk	EMG CCRs	The sEMG parameters or mediolateral-directed CCR results were not significantly changed.
Fantini et al. [72]	Single-hinged brace	12 P (7F/5M)	Immediate effect	Walk	Muscle activation CCRs	Muscle activity and CCRs were significantly reduced.
Hall et al. [21]	Single-hinged brace	16 H (7F/9M)	Immediate effect	Walk	Relative contribution	The average relative contributions of muscles were not significantly changed, but the relative contribution of muscles to the lateral compartment load was increased by 2.35%.
Johnson et al. [32]	Double-hinged brace	10 P (-)	3 months	Walk	Muscle	The mean thigh girth measurement was increased by 1.90 cm.

P: patients; F: females; M: males; H: healthy; (-): not mentioned; EMG: electromyography; sEMG: surface electromyography; CCRs: cocontraction ratios.
